The article "Small-Molecule Quinolinol Inhibitor Identified Provides Protection against BoNT/A in Mice" was retracted in 2013. Reasons: plagiarism; plagiarized text.

# Small-Molecule Quinolinol Inhibitor Identified Provides Protection against BoNT/A in Mice

**DOI:** 10.1371/journal.pone.0047110

**Published:** 2012-10-11

**Authors:** Padma Singh, Manglesh Kumar Singh, Dilip Chaudhary, Vinita Chauhan, Pranay Bharadwaj, Apurva Pandey, Nisha Upadhyay, Ram Kumar Dhaked

**Affiliations:** Biotechnology Division, Defence Research and Development Establishment, Gwalior, Madhya Pradesh, India; Univ of Bradford, United Kingdom

## Abstract

Botulinum neurotoxins (BoNTs), etiological agents of the life threatening neuroparalytic disease botulism, are the most toxic substances currently known. The potential for the use as bioweapon makes the development of small-molecule inhibitor against these deadly toxins is a top priority. Currently, there are no approved pharmacological treatments for BoNT intoxication. Although an effective vaccine/immunotherapy is available for immuno-prophylaxis but this cannot reverse the effects of toxin inside neurons. A small-molecule pharmacological intervention, especially one that would be effective against the light chain protease, would be highly desirable. Similarity search was carried out from ChemBridge and NSC libraries to the hit (7-(phenyl(8-quinolinylamino)methyl)-8-quinolinol; NSC 84096) to mine its analogs. Several hits obtained were screened for *in silico* inhibition using AutoDock 4.1 and 19 new molecules selected based on binding energy and Ki. Among these, eleven quinolinol derivatives potently inhibited *in vitro* endopeptidase activity of botulinum neurotoxin type A light chain (rBoNT/A-LC) on synaptosomes isolated from rat brain which simulate the *in vivo* system. Five of these inhibitor molecules exhibited IC_50_ values ranging from 3.0 nM to 10.0 µM. NSC 84087 is the most potent inhibitor reported so far, found to be a promising lead for therapeutic development, as it exhibits no toxicity, and is able to protect animals from pre and post challenge of botulinum neurotoxin type A (BoNT/A).

## Introduction

Botulinum neurotoxins (BoNTs), produced by *Clostridium botulinum*, *C. baratii* and *C. butyricum*, consist of seven immunologically distinct serotypes (A–G) are the causative agents of a life-threatening neuroparalytic disease known as botulism. The potency, longevity of BoNT intoxication has facilitated use of BoNTs as therapeutic agents [1], [2], [3], [4], [5] and the ease with which these toxins can be produced make them potential bioweapons and bioterrorism agents [6], [7]. Overdose with BoNT therapeutics can also result in systemic botulism [8]. BoNTs are the only toxin group in the six most dangerous biothreat agents (Category A agents) listed by Centers for Disease Control and Prevention (CDC) (http://www3.niaid.nih.gov/Biodefense/bandc_priority.htm). BoNTs are synthesized as ∼150-kDa single-chain protoxins that are post translationally processed by proteolytic cleavage to form a disulfide-linked dimer, composed of a 100-kDa heavy chain (HC) and a 50-kDa light chain (LC) [9]. The HC comprises a 50-kDa C-terminal domain (Hc) that participates in the binding of toxin to productive ectoacceptors on the cell surface of peripheral cholinergic nerve cells [10] and the 50-kDa N-terminal domain (Hn) of the HC facilitates the translocation of the LC across an endosomal membrane into the cytosol of the nerve cell [11]. The LCs are zinc metalloendoproteases [3.4.24] that exhibit extraordinary specificities for SNARE (soluble N-ethylmaleimide-sensitive factor attachment protein receptor) proteins: SNAP-25, VAMP/synaptobrevin and syntaxin [12], [13], [14], [15]. SNARE proteins are essential for exocytosis of neurotransmitter and cleavage of these protein(s) by BoNT inhibits the release of acetylcholine from synaptic terminals leading to neuromuscular paralysis or botulism [16]. The most effective immunotherapy for protection against BoNTs relies on vaccination with pentavalent toxoid species, although supplies are reserved for high-risk individuals [17]. Moreover vaccination of general public also restricts subsequent BoNT's therapeutic applications, if needed. There are no therapies available for BoNT mediated post neuronal intoxication. The current treatments for BoNT poisoning are limited to: (i) the administration of antitoxin(s) to neutralize and clear toxin from the circulation which is not effective in post neuronal intoxication [6] and, therefore, would be of limited use following an act of bioterror (as it is likely that victims would seek medical attention only after enervation); and (ii) mechanical ventilation which is necessary once BoNT-induced paralysis compromises thoracic muscle contraction. However, the latter form of treatment would also be impractical, even a limited act of bioterror employing BoNT(s), as critical care resources would likely to be overwhelmed. The estimated cost for treating a botulism patient with such intensive care could be as high as $350,000 [18]. Antibody therapy can be very effective; it has several limitations, including limited availability, lot-to-lot potency, variability and short window of application. Thus, the hypothesis rationalizing a small-molecule-based therapeutic approach for the treatment of BoNT/A-LC intoxication is as follows: Small drug like molecules can penetrate into the neuronal cytosol and inhibit the toxin's proteolytic activity during post neuronal intoxication. Alternatively, small-molecule inhibitors of BoNT are sought to antagonize the extracellular or intracellular toxin and can be potentially used to treat pre- and post-exposure. Additionally, if stockpiled in dry, sunlight free, temperature-controlled locations, chemically stable small-molecules would remain viable for many years. In contrast, vaccines possess comparatively shorter self-lives. Moreover, with respect to the development of small-molecule therapeutics, the BoNT/A-LC represents a top priority as it possesses the longest duration of activity in the neuronal cytosol in comparison to other BoNT-LCs known to cause botulism in human [5]. Research efforts to identify antagonists against BoNT intoxication have dramatically increased in recent years. However, the discovery and development of BoNT/A small-molecule inhibitors have been a challenging task for researchers since long. Part of the difficulty in this endeavor can be attributed to the unusually large peptide substrate-enzyme interface [19], [20] that requires a small-molecule with high affinity to effectively block substrate binding [21]. Also, the BoNT and its domains show considerable conformational flexibility, making design of effective inhibitors complicated. Despite these challenges, a number of papers have been published on the initial steps to discover and develop inhibitors of BoNT/A protease activity using different approaches. Using high throughput screening of the NCI Diversity Set as well as a series of 4-aminoquinolines, Burnett et al. [22] identified several small-molecule inhibitors of BoNT/A from which a common pharmacophore was predicted using molecular modeling [23]. Quinolinol derivatives (QAQ, NSC1010 and others) were reported to inhibit BoNT/A as determined by biochemical, cell and tissue based assay [24]. Mechanism of QAQ binding to BoNT/A-LC and mode of inhibition was studied in detail by Lai et al. [25]. Similarly, a high throughput screening of a library of hydroxamates [26] resulted in the selection of 4-dichlorocinnamic hydroxamate as a lead structure for further development [10]. Capkova et al. [27] structurally modified 2, 4-dichlorocinnamic acid hydroxamate to improve its potency. On the other hand, a computational screen of 2.5 million compounds resulted in the identification of an inhibitor with a Ki of 12 µM [28], but this value was later invalidated [21]. Computer-aided optimization of this inhibitor resulted in an analog that showed a two-fold improvement in inhibitory potency and displayed competitive kinetics by chelating the active site zinc atom [21].

Though the above approaches have resulted in the identification of a number of small-molecules as BoNT/A inhibitors, no compound has yet advanced to pre-clinical development [24], [29], [30], [31]. The majority of such molecules reportedly demonstrated to be effective in enzymatic assays [21], [23], [27], [28], [32], [33] and a few small-molecules have been tested in cell-based assays [34], [35], [36], [37]. But the information shows that small-molecules can significantly protect mammals against BoNT/A is scanty [31], [36]. We screened the ChemBridge and NSC libraries, consisting of millions of compounds of unknown function for similarity search to 8-hyroxy quinolinol lead, NSC 84096. Since some of these compounds were commercially available and their functions are currently undefined, we reasoned that novel inhibitors could be identified. Herein we report the effective small-molecule BoNT/A inhibitors with promising *in vivo* pharmacokinetics. Our results demonstrate that small-molecule can protect mice against pre and post BoNT/A challenge and support pursuit of small-molecule inhibitor as a cost effective alternative for treating botulism and for biodefence measures.

## Materials and Methods

### 1. Expression and Purification of Recombinant BoNT/A-LC Protein

Previously, we have reported the conditions for the high level expression and purification of biologically active light chain protein of botulinum neurotoxin type A from a synthetic gene [38]. In brief, full length BoNT/A-LC gene was cloned in pQE30 vector and expressed in *E. coli* SG13009 at 21°C for 18 h. The rBoNT/A-LC was purified using Ni-NTA agarose and analyzed by 12% SDS-PAGE. The purified protein was characterized by western blotting and MALDI-TOF. The rBoNT/A-LC was dialyzed against 20 mM HEPES (pH 7.4) containing 200 mM NaCl, 10% glycerol (v∶v), pH 7.4 and stored at −20°C until used.

### 2. Assay of rBoNT/A-LC Activity on Synaptosomes

#### 2.1. Preparation of Rat Brain Synaptosomes

Crude synaptosomes were prepared from rat brain as described by Ferracci et al. [39]. Briefly, fresh rat brain (1 g) was homogenized with a teflon homogenizer in 10 ml of chilled homogenization buffer (0.32 M sucrose, 1 mM PMSF, 1 mM EDTA, and 10 mM HEPES, pH 7.5). Homogenized sample was centrifuged at 10,000 rpm for 15 min at 4°C, and supernatant (∼2 mg/ml) was collected and filtered with a 0.22 µ membrane and stored at −20°C.

#### 2.2. Optimization of Assay

The cleavage reaction was optimized with respect to concentrations of synaptosome substrate and rBoNT/A-LC, incubation time, and composition of cleavage buffer. Catalytic activity of rBoNT/A-LC protein was performed in 50 µl reaction mixture containing varying concentrations of rat brain synaptosomes and rBoNT/A-LC in reaction buffer (25 mM Tris, 100 mM NaCl, 19.2 mM glycine, 100 µg/ml BSA, 0.1 mM DTT, 10 µM ZnCl_2_, pH 7.5) and incubated at 37°C. For the time course analysis the reactions were stopped by adding 4× SDS-PAGE sample buffer at 1, 2, 5, 10, 20, 30, 60, 120, 180, 240, 300, 360, 420 and 480 min. The samples were analyzed by western blotting.

### 3. Molecular Docking Studies

#### 3.1. Preparation of Ligands and Receptor

The NCI and ChemBridge database libraries were chosen for virtual screening of small-molecule inhibitors on the basis of structure similarity searches. The structures of selected molecules were drawn by Chemsketch (ChemDraw) software (http://www.acdlabs.com) and saved as MDL mol files. The energy minimized pdb files were generated using ArgusLab 4.0.1 (http://www.arguslab.com). Ligand files in the pdb format were opened in AutoDock (4.1) for preparation. Once opened, ligand files were edited and saved in pbdqt format. The three-dimensional structure of BoNT/A-LC (PDB code 3BON) was obtained from the RCSB Protein Data Bank. All water molecules except those which participate in catalysis were removed. The rigid and flexible residues of the protein were selected, and two additional files were created; a file 3BONrigid.pbdqt and file 3BONflex.pbdqt.

#### 3.2. Grid Generation and Running AutoGrid

AutoDock requires pre-calculated grid maps, one for each atom type present in the ligand being docked. AutoGrid 4.1 was used to create autogrid .gpf, .glg, .fld and map files of atoms for protein. The Grid box was constructed around the active site residue Glu262 which plays a pivotal role in the catalytic activity of BoNT/A endopeptidase [40], [41]. The active site residues that surrounded by docking box were Phe163, Gln162, Glu164, Cys165, Lys166, Phe194, Glu224, His227, Arg231, Ala236, Ile237, Pro239, Val258, Ser259, Glu261, Arg363, Tyr366, and Zn(II).

#### 3.3. Preparing the Docking Parameter File and Running AutoDock

The final step in submitting the docking was to run the AutoDock function. To prepare this, the protein's rigid pbdqt file, the flexible pdbqt file and ligand's pdbqt file were specified. At the end of a docking process, the output file ‘.dlg’ showed the docked conformations. These conformations were compared one to another to determine similarities and they were clustered accordingly. The root mean square deviation (RMSD) was used to determine whether two docked conformations are similar enough to be in the same cluster. After that these clusters were ranked from the lowest energy to highest.

### 4. Screening of Inhibitors using Rat Brain Synaptosome

Test compounds were obtained from the Drug Synthesis and Chemistry Branch, Developmental Therapeutics Program, Division of Cancer Treatment and Diagnosis, NCI (Bethesda, MD) and ChemBridge Corporation (San Diego, CA). BoNT/A peptide inhibitor (RRGC) was purchased from Bio Basic (Ontario, Canada). Compounds selected after virtual screening were tested in cleavage-based rBoNT/A-LC enzymatic assay. The inhibitors were dissolved in absolute DMSO and stock solutions were made up to 20 mM.

Initial screening was performed in 40 µl reaction mixture containing 2.05 µg synaptosomes and 6 µM rBoNT/A-LC in cleavage buffer along with the 1 mM small-molecules. For determination of inhibitory molar ratios of small-molecules to rBoNT/A-LC, different concentrations of the small-molecules (100, 200 and 500 µM) and rBoNT/A-LC (25 pM, 200 nM and 6 µM) were used. In control assays, positive control was accomplished without test compound and rBoNT/A-LC and negative control test compound was replaced by DMSO. The incubation was carried out at 37°C for 15 min. The reactions were stopped by adding 4× SDS-PAGE sample buffer followed by heating at 100°C for 5 min.

### 5. Determination of the IC_50_

Fifty-percent inhibitory concentration (IC_50_) values for rBoNT/A-LC were calculated from nine concentrations of compound via dose-response measurements. The reactions were set up in duplicate as described earlier with the decreasing concentrations of inhibitors, keeping the concentration of rBoNT/A-LC constant at 10 nM. Each value is the average of two independent determinations. In all the cases, standard deviations were less than ±20%.

### 6. Western Blot Analysis

Proteins from catalytic reactions were separated on a 13% SDS-PAGE before transfer to a 0.2 µ nitrocellulose membrane for 60 min at 100 V. After blocking in 5% skim milk/PBS for 2 h at room temperature (RT), the membrane was washed three times for 5 min at room temperature with PBST [2 mM Phosphate buffer (pH 7.4), 137 mM NaCl, 2.7 mM KCl, and 0.1% Tween 20(v/v)]. Rabbit anti-SNAP-25 antibody against N-terminal SNAP-25 protein (Sigma, USA) was added at the dilution of 1∶5000 in PBS and the blot was incubated for 1 h at RT and washed four times with PBST. Goat anti-rabbit HRP conjugate antibody at a dilution of 1∶30000 into PBS was added and further incubated for 1 h at RT. Membrane was again washed with PBST four times, each of 10 min. Bound antibodies were detected by chemiluminescence using an ECL western blot kit (Biological Industry, Israel) as per manufacturer's instructions. Film was exposed for 15 s before development. The inhibitory action (%) of the molecules was evaluated by densitometric analysis of blots using GS800 densitometer and Quantity One software (BioRad, USA).

### 7. Evaluation of Small-molecule Inhibitors in Mouse Model

Four inhibitor molecules were selected for *in vivo* experiment based on *in vitro* results. Female Balb/c mice (20–25 g weight) were used for *in vivo* experiments and they were divided into seventeen groups having five mice each (four groups for each molecule and one group for BoNT/A control). Mice from one group received 5LD_50_ of BoNT/A (in 200 µl PBS) intraperitoneally (ip). All four compounds were tested using four groups of mice as described below. To determine the toxicity of compounds, each of the molecule (1 mM) solubilized in PBS/DMSO (9∶1) was injected per mouse ip in second group. In third group, 100 µl (1 mM) of small-molecule inhibitor mixed with 5 LD_50_ of BoNT/A holotoxin was injected ip. Fourth group received 5 LD_50_ of BoNT/A, 30 min before the inhibitor injection. In last group of animal (fifth group) 100 µl each (1 mM) of small-molecules were injected 30 min prior to challenge with 5 LD_50_ of BoNT/A. All mice were examined for 4 days at hourly interval for survival, behavior, breath, and extraocular symptoms of botulism. All the animal experiments were approved by the Laboratory Ethical Committee on Animal Experimentation of Defence Research and Development Establishment, Gwalior, India via permission no. BT/01//DRDE/2009 and all efforts were made to minimize suffering.

## Results and Discussion

In the wake of the events of September 11, 2001, research efforts aimed at the discovery of potent antagonists for agents of bioterrorism have increased exponentially. However, despite the plethora of new data that has emerged in the past 5 years, an established pharmacophore validated through *in vivo* models of exposure remains elusive. Indeed, in the case of BoNT, few studies have reported the assessment of any small-molecule antagonist in animal models [31], [36]. The development of small-molecule inhibitors as intraneuronal therapeutics is a crucial unmet need. Our initial impetus for producing recombinant LC as a reagent to be utilized in synaptosome based assay for the screening of potential inhibitors of the BoNT/A-LC protease activity. A 1401 bp DNA fragment encoding BoNT/A-LC along with 14 amino acids of translocation domain and 15 amino acids of N-terminal heavy chain was selected to produce rBoNT/A-LC as already reported in our previous study [38].

### 1. Strategy and Virtual Screening

We focused on serotype A since it is the most prevalent and well-studied among the various serotypes in human intoxication. We used *in silico* screening to identify BoNT/A inhibitors. The ChemBridge and NSC libraries, consisting of millions of compounds of unknown function, were chosen for virtual screening to chemoinformatically “mine” novel small-molecule non-peptidic inhibitors (SMNPIs). Since some of these compounds were commercially available and their functions currently undefined, we reasoned that novel inhibitors could be identified.

Peptidomimetics and hydroxamic acid-based inhibitors have been developed that display inhibitory effects in the high nM range for the light chain of the BoNT serotype A (BoNT/A -LC) [26], [34], [35], [40], [42], [43]. Compounds that contain zinc-coordinating sulfhydryl moieties might potentially inhibit host zinc proteases thereby making them poor therapeutic leads. The characteristically poor pharmacokinetics of hydroxamates, their instability, and their reported toxicity, which is likely due to their inhibition of an array of metalloproteases, also make them problematic as therapeutic agents [44], [45]. We focused on the 8-hydroxy quinolinol lead NSC 84096 for database search. Selection of this compound was based on: (i) NSC 84096 is reported to be very potent and serotype A selective inhibitors [24]; (ii) it is reported to be non toxic and active in cell based and mouse phrenic nerve hemi-diaphragm (MPNHD) assays [24]; (iii) there are quinolinols in clinical trials for Alzheimer's disease and cancer [46]–[48]; and (iv) quinolinol-based drugs such as linolasept and vioform (generic name: Clioquinol) are available in the market. The compounds from the NCI database were docked into the active site in one of the three dimensional structure of BoNT/A-LC (PDB code: 3BON) [41] after removing the peptide occupying the active site. The top scoring 100 compounds were evaluated in detail; the list was narrowed to 25 compounds (based on binding energy and K_i_) that interacted well with the active site Zn and demonstrated a ‘good fit’ in the BoNT/A-LC binding site (Table S1). Among these, twelve compounds were studied in detail and *in silico* parameters obtained were summarized in table 1. Other thirteen molecules were not available for the *in vitro* and *in vivo* studies.

**Table 1:** *In silico* docking parameters obtained for selected Quinolinol derivatives used in the study by AutoDock 4.1.

S No	Compound ID	Ki (nM)	Binding energy	Number of interactions	Interaction between	Vdw_hb_ desolve energy	Electrostatic energy	Total internal energy	Torsional energy	Ref RMS
1	CB6377128	539.2 pM	−12.64	32	ASP203:N1, GLU197:N1(OH), LEU367:N1(S), Tyr366:OH, Phe163:NH	−7.18	−0.06	−2.84	1.37	14.89
2	CB7969312	28.3	−10.3	1	TYR366-OH	−8.66	−0.11	−2.78	1.92	11.79
3	CB7967495	4.26	−11.42	1	LYS166-N of C6H6	−6.75	−0.16	−2.3	1.65	14.92
4	CB7925339	1.04	−12.25	1	GLU262-OH	−7.74	−0.12	−2.14	1.92	19.46
5	CB7887535	3.63	−11.51	1	TYR366-OH	−7.47	−0.03	−2.04	1.37	12.04
6	CB6378306	6.07	−11.21	2	LYS166:O-CH3	−6.36	−0.17	−2.05	1.92	17.13
7	CB6376015	76.61	−9.71	5	THR365:N0,N1,O1(3)	−7.38	−.05	−2.57	1.1	16.48
8	NSC1010	22.36	−10.44	1	GLU262-NH	−7.08	−0.86	−2.72	1.37	10.85
9	NSC84090	2.11	−11.83	1	Glu164-NH	−6.7	−0.06	−2.23	1.37	10.96
10	NSC84096	25.09	−10.37	1	Glu164-NH	−8.18	0.14	−3.05	1.1	13.5
11	NSC84087	52.95	−9.93	1	Glu164-NH	−6.72	0.03	−3.18	1.37	12.87
12	NSC84093	145.66	−9.33	2	Glu266-NHCys165-OH	−6.67	−0.04	−3.0	1.37	16.01

The particular class of quinolinol identified in our study is reported to specifically inhibit BoNT serotype A and does not inhibit simply by chelating active-site zinc. The structures of the quinolinol derivatives under investigation contain additional basic moieties including 2-amino or 3-amino pyridine (Table S1). The presence of these structural motifs suggests that these molecules may interact with the hydrophobic pocket located in the active site of the BoNT/A-LC and interact with Tyr366 and Val258. The quinolinol moiety alone in the presence of zinc does not inhibit the proteolytic activity of BoNT serotypes A and B as described by Adler et al. [49]. Data obtained from *in silico* docking along with the *in vitro* inhibition at 100 µM concentration of quinolinol derivatives used in the study is summarized in table S2. As shown in figure 1, NSC 84087 is docked in the large hydrophobic pocket of the BoNT/A-LC active site, and its hydroxy quinoline moiety coordinates with zinc. The methoxy group of aniline ring can form a hydrogen bond with His227, which coordinates with zinc, and may contribute to the specificity and potency of this inhibitor. Additionally, the phenyl group is found to fit between Glu164 and Cys165 which are reported to participate in substrate binding [40]. This could explain the importance of hydroxy group in inhibiting BoNT/A-LC, and suggests that the quinolinols inhibit BoNT/A by blocking the active site zinc. It should be noted that the crystal structures of the complexes of known small-molecule and peptide inhibitors with BoNT/A-LC have shown that chelation to zinc is involved in the binding and inhibition of the light chain in both cases [40], [41].

**Figure 1:** Binding mode of NSC84087 into BoNT/A-LC substrate binding cleft showing ligand (grey) interacting with Zn atom (green) and other amino acids (ie HIS 227, GLU 164 and GLU 262).

### 2. Inhibition of rBoNT/A-LC using Synaptosome Model

BoNT-LCs are remarkable among proteases for the extremely long substrate required for efficient proteolysis, whereas other microbial metalloproteases have been found to display activity against as short as dipeptides [50]. The catalytic LC domain of BoNT/A is a compact globule consisting of a mixture of α-helices, β-sheets, and α -strands with a zinc-containing metalloprotease active site bound deeply inside a large open cavity [19]. The remarkable substrate selectivity of BoNT/A for SNAP-25 has been explained to be a consequence of extensive interactions with two exosite domains distinct from the active site [51]. A model for substrate recognition has been proposed in which α-exosite binding occurs first via helix formation in the appropriate region of SNAP-25, followed by β-exosite recognition and subsequent conformational changes in the enzyme to facilitate efficient substrate cleavage [19]. This model argues that, without exosite binding, BoNT/A-LC is a significantly less efficient enzyme, and thus these regions could be targeted for lead development. BoNT/A-LC requires a minimal SNAP-25 peptide sequence of ∼51 amino acids to achieve efficient cleavage, and optimal binding occurs with only the full length SNAP-25 [50]. The crystal structure of SNAP-25 (residues 141–204) bound to BoNT/A-LC (residues 2–420 with active site mutations E224Q, Y366F) provides an explanation for this finding as binding involves protein exosites that anchor the substrate and position the scissile bond for cleavage [19]. BoNT/A-LC recognizes multiple sites within SNAP-25; an extended surface on SNAP-25 distanced from the site of cleavage [19], [50] and residues adjacent to the scissile bond that are discontinuous and appear as pockets surrounding the cleavage site [51]. This implicates multistep recognition of SNAP-25 for cleavage by BoNT/A-LC. Intracellular BoNT/A-LC is shown to directly bind SNAP-25 on the plasma membrane. Solid phase binding showed that the N-terminal residues of BoNT/A-LC bound residues 80–110 of SNAP-25, which was also observed in cultured neurons. Association of the eight N-terminal amino acids of BoNT/A-LC and residues 80–110 of SNAP-25 also enhanced substrate cleavage by 2 folds. Two regions (80–110) and (180–197) of SNAP-25 contribute to the high affinity binding to BoNT/A-LC [20].

The LC of BoNT/A specifically cleaves the C-terminal 9 amino acids residues of SNAP-25, between residues Gln197 and Arg198 of the 206, thereby producing a 24 kDa cleaved protein [12]. Analytical techniques have been developed that directly assess SNAP-25 cleavage in cell lysates by immunoelectrophoresis [39]. We analyzed the amount of intact versus cleaved SNAP-25 western blotting to determine BoNT/A-LC activity/inhibition using rat brain synaptosomes.

Screening was conducted by using a recombinant catalytic light chain of BoNT/A, produced in a soluble and stable form that can be easily expressed in *E. coli* at high levels and purified in large quantities necessary for screening. The extent of cleavage of SNAP-25 in synaptosomes by rBoNT/A-LC was determined by western blot analysis using monoclonal antibodies against SNAP-25. The selected compounds were initially screened for inhibition of rBoNT/A-LC mediated cleavage of synaptosomal SNAP-25 isolated from rat. NSC 84090 and Tetra peptide inhibitor RRGC were not showing any inhibition, however complete inhibition was recorded with 100 µM of CB796312, CB7925339, CB7887535, CB6378306, CB6376015, CB6377128, NSC84096, like other previously reported compounds NSC 1010 and NSC 84096 as shown in the figure 2. Whereas CB7967495 & NSC84093 showed decrease in inhibition (87 and 85% respectively) of endopeptidase cleavage of SNAP 25 using the same concentrations of rBoNT/A-LC (200 nM). From this experiment seven new lead analogs (CB796312, CB7925339, CB7887535, CB6378306, CB6376015, CB6377128, NSC84096,) at 100 µM were found to be exhibited complete protection of rBoNT/A-LC (200 nM) mediated SNAP-25 cleavage. Among these seven new molecules, five compounds (CB7925339, CB7887535, CB6378306, CB6376015 and NSC 84087) showed near-complete to- complete inhibition of SNAP-25 cleavage at 10 µM, while CB796312 afforded only 78% protection (Fig. 3). Surprisingly remaining one molecule CB6377128 did not show any significant inhibition of endopeptidase activity at 10 µM (Fig. 3) whereas it had shown protection at 100 µM (Fig. 2). The molecule NSC 84093 showed again decrease in protection from 85% at 100 µM (Fig. 3) to 58% at 10 µM (Fig. 2).

**Figure 2:** Initial screening of different compounds by western blotting using specific antibodies. RRGC and twelve other compounds (CB7969312, CB7967495, CB7925339, CB7887535, CB6378306, CB6376015, CB6377128, NSC1010, NSC84096, NSC84090, NSC84087 and NSC84093 were tested for their inhibition activity. To determine inhibition activity of these compounds, 2.05 µg synaptosomes prepared from rat brain was incubated with 200 nM of rBoNT/A-LC and 100 µM of each compounds solubilized in DMSO at 37°C for 15 min as described in materials and methods. Proteins were visualized using appropriate HRP-labeled second antibody by ECL. Nine molecules (CB796312, CB7925339, CB7887535, CB6378306, CB6376015, CB6377128, NSC1010, NSC84096, and NSC84087) showed complete inhibition while CB 7967495 & NSC84093 showed 87 and 85% of inhibition respectively. Significant inhibition was not observed with RRGC and NSC 84090 molecules.

**Figure 3:** Determination of inhibition activity of eight selected compounds at 10 µM. In this experiment, reaction without inhibitor was used as a negative control and with RRGC (known inhibitors) for comparison. Near complete to complete inhibition of rBoNT/A-LC endopeptidase activity was observed by CB7925339, CB7887535, CB6378306, CB6376015 and NSC 84087 molecules. NSC 84093 and CB796312 showed 58 and 78% inhibition, respectively. No inhibition was observed with compound CB 6377128.

As shown in figure 4, NSC84087 showed dose dependent inhibition of endopeptidase activity of rBoNT/A-LC (10 nM), the IC_50_ is estimated to be 40 nM (±3.7 nM). This indicates that 50% BoNT/A-LC inhibition is achieved when the inhibitor: rBoNT/A-LC molar ratio is 4∶1; however 100% inhibition was recorded at 6∶1 molar ratio. The extent of inhibition and the IC_50_ values of these leads were comparable to or even better than those of previously reported small-molecule inhibitors [(10000∶1) Park et al. [28]; (3000∶1) Burnett et al. 2007 [35]; (800∶1) Tang et al. 2007 [21]; (150∶1) Eubanks et al. 2007 [36]; (320∶1) Cai et al. 2010 [52]; (2000∶1) Pang et al. 2010 [31]; (3000∶1) Ruthel et al. 2011 [37]; (250∶1) Burnet et al. 2010 [32]; (350∶1) Thomson et al. 2011 [53], molar ratios given in parenthesis are of inhibitor: BoNT/A-LC]. The molar ratio between inhibitor and BoNT/A-LC molecules at 50% inhibition provides better parameter for comparison between assays, since it normalizes the neurotoxin used. The lower molar ratio in synaptosome based assay reflects the inhibitor's efficiency is more relevant to *in vivo* conditions. In fact, the IC_50_ values of the compounds increased (worsened) 4- to over 50-fold when the concentration of one of the model enzymes, *β*-lactamase, was increased 10-fold, from 1 nM to 10 nM [54]. The authors also suggested for the unifying mechanism to be followed for the discovery of the inhibitors.

**Figure 4:** Western blot showing dose dependent inhibition of rBoNT/A-LC endopeptidase activity by NSC 84087. Three different concentrations (10, 1 and 0.10 µM) of NSC 84087 molecule were incubated separately with 10 nM of rBoNT/A-LC and 2.05 µM of rat brain synaptosomes at 37°C for 15 min as described in materials and methods. Complete inhibition was observed at 10 and 1.0 µM. Results from Western blots are representative of two independent preparations. DMSO was used in one of the reaction to observe the effect of solvent on the inhibition.

Major advantages of a synaptosome based assay are: (i) it provides full length SNAP-25 substrate to β-exosite recognition and subsequent conformational changes in the enzyme to facilitate efficient substrate cleavage. It has been considered that, without exosite binding, BoNT/A is a significantly less efficient enzyme; and (ii) it simulates the microenvironment of the neurons. The other advantages are considerable reduction in the number of animals used (millions of reactions can be performed from synaptosomes isolated from single rat brain), substrate stability (synaptosomes isolated are stable for use as substrate for more than year), instrumentation requirement and cost incurred, especially when used for assessing large numbers of target molecules.

We suspect the use of small peptide substrates (∼17mer peptides/fluorescent substrate which is minimum substrate required for BoNT/A) in high-throughput screening and identification of small-molecule inhibitors is the reason for *in vitro* and *in vivo* disconnect which is reported by Eubanks et al. [36]. In majority of such studies carried out for the development of small-molecule inhibitors against botulinum neurotoxins, higher potency of small-molecule inhibitors observed during evaluation in the *in vitro* assay systems using small peptide substrate, may have resulted due to the suboptimal activity of BoNT/A-LC. As these small substrate peptides used for *in vitro* screens are not long enough to simultaneously occupy cleavage site and either of the exosite, hence it is clear inhibition in fluorescent peptides based assays relies on the interactions in the enzyme active site. However, our findings argue that in the context of BoNT therapeutics, caution should be used in extrapolating *in vivo* potency from these assays.

### 3. Evaluation of Small-molecule Inhibitors in Mouse Model

To be useful as therapeutics, the newly identified inhibitors must: (i) be able to enter neurons; (ii) inhibit the toxin within the neuronal cytosol; and (iii) be tolerated by animals (*i.e.* possess acceptable toxicity profiles). A true test or ultimate goal for inhibitors evaluated in both cell-free systems and even for cell based assays is whether their effectiveness holds true *in vivo*. The effectiveness of small-molecule inhibitors in the *in vitro* and *ex vivo* assays was only demonstrated when the compound was premixed with BoNT/A; thus far, pre-loading the inhibitor did not protect cells/tissues against BoNT intoxication [24]. The small-molecule inhibitor that was reported to be active in primary neurons [22] was demonstrated to show a dose-dependent inhibition of SNAP-25 cleavage in a non-pre-loading system (cells were pretreated with inhibitor for 45 minutes followed by incubation with BoNT/A in the continuous presence of inhibitor). Additionally, the inhibitors reported by Eubanks et al. [36] and Boldt et al. [34] were characterized in cell culture assays that involved mixing BoNT/A toxin and varying concentrations of inhibitor. To our knowledge, no group has been able to provide experimental evidence showing that their inhibitors work in a pre-loading system.

After completion of our *in vitro* screening, three compounds were deemed to have suitable activity and were advanced into animal models (CB 7887535, CB6378306 and NSC 84087). The fourth compound, included for comparison, was a molecule previously well characterized and reported to inhibit specifically BoNT/A-LC (NSC 1010). To examine the lead compounds *in vivo*, a well-established mouse bioassay was used. This model is the Food and Drug Administration (FDA) standard for assessing BoNT levels and the universally accepted method for the study of BoNT antagonists (e.g., antibodies, small-molecules) [55]. For evaluation of inhibitory potential of small-molecules, they were injected into test animals as described in materials and methods. All animals were monitored continuously for a period of 4 days for signs of botulism, and the time of death was recorded. Of the compounds studied, one compound (NSC 84087) showed efficacy in preventing BoNT/A-induced death in all three modes of injections and an injection dosage of 100 µl of 1 mM per animal survived the BoNT challenge with no obvious signs of botulism upto 20 h (Fig. 5). All the mice of inhibitor followed by BoNT/A group, showed symptoms after 20 h and died within 30 h of injection. Mice of other two groups, BoNT/A followed by inhibitors and inhibitors toxin premixed, survived upto 48 h. In similar *in vivo* studies, conducted by Eubanks et al. [36] and Pang et al. [31] reported mere 36% increase time to death and 10% of mice survival after days of standard observation period, respectively. The second compound CB 7887535 extended the time to death from ∼9 to ∼20 h, corresponding to a more than 100% increase in time to death. Although this appears modest at first glance but this enhancement is also remarkable considering potency of the neurotoxin. In contrast, animals treated with NSC 1010 and CB6378306 molecules at similar doses died without any statistically significant increase in the time to death relative to control group (between 8–10 h). In all cases, no toxicity was observed from treatment with either inhibitor compound alone.

**Figure 5:** *In vivo* evaluation of selected small-molecules in mouse model against 5LD_50_ of BoNT/A. NSC 1010 and CB6378306 were found incapable in inhibiting BoNT endopeptidase activity in mouse as a result of which animals treated with these groups died along with control (mice treated with 5LD_50_ of BoNT/A only), although mice treated with CB 7887535 molecules resulted in extended survival time from ∼9 h to ∼20 h. The group of animals either treated with 5LD_50_ of BoNT/A followed by NSC84087 molecules or treated with the mixture of NSC84087 & 5LD_50_ of BoNT/A showed survival upto 48 h. Results are expressed as an average of three independent experiments ± s.d.

### Summary

Rat brain synaptosome model has been used to *in vitro* screen small-molecule inhibitors which can more accurately predict in vivo efficacy. Using this model, five highly potent non-toxic BoNT/A small-molecule inhibitors have been identified in present study. These compounds effectively inhibited the protease activity rBoNT/A-LC and the compound NSC 84087 is able to protect against BoNT/A challenge and encourages the pursuit of small-molecule BoNT inhibitors for the development of next generation botulism therapeutics. We recognize that these leads are viable drug candidates, and, they need to be optimized for other important drug characteristics including absorption, distribution, metabolism, excretion and toxicity (ADMET) for further clinical use.

## Supporting Information

Table S1 List of compounds selected based on similarity search (1–20 New leads and 21–25 reported molecules) with binding energy and Ki obtained by docking.
(DOC)

Table S2 Structural formula and results of initial screening at 100 µM of small-molecules on synaptosome against recombinant full-length BoNT/A light chain (200 nM).
(DOC)
